# Analysis of Molecular Mechanism of YiqiChutan Formula Regulating DLL4-Notch Signaling to Inhibit Angiogenesis in Lung Cancer

This article has been retracted.

**DOI:** 10.1155/2021/8875503

**Published:** 2021-02-12

**Authors:** Jiayin Li, Rui Han, Jing Li, Linzhu Zhai, Xinying Xie, Jing Zhang, Yao Chen, Jiamin Luo, Sisi Wang, Zhe Sun, Yang Cao, Lizhu Lin, Qiuye Yang

**Affiliations:** ^1^Cancer Center, The First Affiliated Hospital to Guangzhou University of Chinese Medicine, Guangzhou 510405, China; ^2^Department of Oncology, The First Affiliated Hospital to Hunan University of Chinese Medicine, Changsha 410000, China; ^3^Department of General, The First Affiliated Hospital to Guangzhou University of Chinese Medicine, Guangzhou 510405, China; ^4^The First Affiliated Hospital to Guangzhou University of Chinese Medicine, Guangzhou 510405, China; ^5^Department of Medical Technologic, The First Affiliated Hospital to Guangzhou University of Chinese Medicine, Guangzhou 510405, China

## Abstract

In order to explore the specific mechanism of YiqiChutan formula (YQCTF) in inhibiting the angiogenesis of lung cancer and its relationship with delta-like ligand 4- (DLL4-) Notch signaling, 30 healthy BALB/c-nu/nu rats were selected and divided into three groups: A549 group (implanted with lung adenocarcinoma cell line A549), NCI-H460 group (implanted with human lung large-cell carcinoma cell line NCI-H460), and NCI-H446 group (implanted with human lung small cell carcinoma cell line NCI-H446) for constructing lung cancer transplanted tumor models. After modeling, the group treated with normal saline was taken as control group, 200 mg/kg of YQCTF was adopted for intervention, and the tumor volume and growth inhibition rate were compared with the vascular targeted inhibitor Sorafenib. HE staining, CD31 fluorescent antibody staining, and microelectron microscopy were adopted to observe the neovascular endothelial cells of the transplanted tumor. The expression of VEGF, HIF-1*α*, DLL4, and Notch-1 in the transplanted tumors in each group was detected by Western blot and RT-PCR at the protein level or mRNA level. Compared with the control group, the YQCTF-treated group had obvious inhibitory effect on lung cancer transplanted tumor and lung cancer angiogenesis. In the YQCTF-treated group, the density of angiogenesis decreased significantly and the vascular lumen structure also decreased, and the expression levels of VEGF, HIF-1*α*, DLL4, and Notch-1 in the YQCTF-treated group were all lower than those in the control group. YQCTF could inhibit the growth of lung cancer transplanted tumor through antiangiogenesis, and it could also reduce the amount of angiogenesis in lung cancer transplanted tumor. In addition, the generation of lumen structure was also hindered, which was realized through the VEGF signaling pathway and DLL4-Notch signaling pathway.

## 1. Introduction

With the development of modern society, environmental pollution and radiation increase people's risk of cancer, which has now become the leading cause of death of Chinese and a major public health problem. Among them, lung cancer is one of the most common cancers. It mostly occurs in people over 40 years old, especially those between 60 and 79 years old. The male to female ratio is 2.3 : 1. Among the deaths of men in at least 35 countries around the world, lung cancer ranks first. Lung cancer remains the leading malignancy in morbidity (11.6%) and mortality (18.4%). As one of the most common cancers, lung cancer is also the leading cause of cancer-caused death [1–3]. At present, the treatment for cancer mainly includes surgery, chemoradiotherapy, and targeted therapy, but these treatments all have serious postoperative complications. The side effects of chemoradiotherapy even directly affect the postoperative survival and life of patients [4]. Current medical research showed that angiogenesis was one of the main mechanisms for tumor growth, metastasis, and invasion. Tumor blood vessels provided nutrition and waste metabolism pathways for tumors, which were key steps and necessary conditions for tumor genesis and metastasis. Therefore, inhibition of tumor angiogenesis has become an important target for clinical treatment of tumors [5, 6]. The YQCTF is an empirical prescription for tumor treatment, composed of rhizoma pinellinae praeparata, Indian Iphigenia Bulb, Gen-Seng, and thunberg fritillary bulb, which cures both symptoms and origins, and it not only benefits “qi” and removes phlegm but also has certain detoxication effect. Chen et al. treated 55 advanced NSCLC patients with YQCTF combined with drugs. The results showed that TCM combined with chemotherapy could better alleviate the clinical symptoms of patients (82.1% vs. 66.7%, *P* < 0.05) and improve the quality of life (82.2% vs. 55.5%, *P* < 0.01) than chemotherapy alone. The objective response rate of tumor was increased (64.3% vs. 29.6%, *P* < 0.01), and there was no statistical difference in peripheral blood cells (*P* > 0.05), suggesting that YQCTF can improve the efficiency and quality of life of elderly patients with advanced NSCLC chemotherapy. In addition to YQCTF combined with chemotherapy, in combination with local therapy, Zhang treated 90 patients with advanced lung cancer by YQCTF combined with radiofrequency ablation, who were divided into TCM group, radiofrequency ablation group, and comprehensive treatment group, with 30 cases each. The results showed that YQCTF could improve the quality of life of patients with radiofrequency ablation by improving patients' functional status, physical status, and lung cancer-specific modules (*P* < 0.05). The efficacy of the combined treatment group was better than that of the traditional Chinese medicine group alone and the radiofrequency ablation group alone (*P* < 0.05). In improving the quality of life and reducing adverse reactions of chemotherapy in patients with advanced lung cancer, Zhang classified 60 cases of stage III and stage IV NSCLC patients into traditional Chinese medicine, western medicine group, and Chinese and western medicine group, each with 20 cases. The FACT-L scale was adopted to analyze patients regarding physical status, relationship with doctors, social/family status, functional status, emotional status, and additional status. The results suggested that YQCTF could not only reduce the toxic and side effects of chemotherapy (*P* < 0.05), but also significantly improve the quality of life of patients (*P* < 0.05). The above experiments indicated that YQCTF has favorable clinical effect on lung cancer and other malignant tumors. Preclinical trials showed that it had a good clinical effect on malignant tumors such as lung cancer [7–9]. However, at present, the inhibitory mechanism of YQCTF for lung cancer is still unclear. Combined with other existing studies, it was speculated that the possible mechanism included inhibition of tumor angiogenesis, inhibition of tumor cell proliferation, induction of tumor small differentiation and apoptosis, and reduction of telomerase activity [10, 11].

In this study, different types of human lung cancer transplanted tumor models were established to explore the effects of YQCTF on the growth and angiogenesis of lung cancer. The expression levels of DLL4 and Notch were measured to further determine whether the inhibitory effect of YQCTF on growth and angiogenesis of lung cancer could be realized through DLL4-Notch signaling pathway, so as to provide a theoretical basis for elucidating the anticancer mechanism of YQCTF in lung cancer.

## 2. Materials and Methods

### 2.1. Experimental Animals and Cells

30 healthy BALB/c-nu/nu nude rats were selected, all of which were healthy males, aged 5-6 weeks, weighing 20-30 g, and with an average weight of 26 ± 4 g (Sun Yat-sen University Laboratory Animal Center). The mice were kept in a clean environment without specific pathogens, with room temperature at around 25°C, and relative humidity at around 60%. The mice were allowed to eat and drink freely, so that they could adapt to the environment in one week.

NSCLC cell lines A549 (adenocarcinoma) and NCI-H460 (large-cell carcinoma) were purchased from the Cell bank of Shanghai, Chinese Academy of Sciences, and SCLC cell line NCI-H446 (small-cell carcinoma) was purchased from the American Type Culture Collection (ATCC). The above cell lines were frozen and stored at -80°C for usage before the experiment.

### 2.2. Cell Culture, Transplantation Tumor of Lung Cancer Model Construction, and Grouping

A549, NCI-H460, and NCI-H446 cells were taken out and quickly melted in warm water at 40°C. The cryopreserved tube was wiped with 75% ethanol on the sterile operating table before opened, more than 10 mL of preheated cell culture medium was added to 25 cm^2^ culture bottle, 10% fetal bovine serum was added to the culture medium, 1 mg/L penicillin and streptomycin were added, and the culture was conducted at 37°C and with 5% CO_2._

The above logarithmic growth cells were collected and resuspended to serum-free medium, with the final cell concentration maintained at 5.0 × 10^7^ cells/mL. Subcutaneous inoculation was performed on the right back of each nude rat, and 0.2 mL cell suspension was administered to each nude rat (the three groups were, respectively, inoculated with A549, NCI-H460, and NCI-H446 cells). After inoculation, the daily behavior of the animals was observed. Meanwhile, the length and width of the tumor were calculated with vernier caliper the day after inoculation. The tumor volume was calculated and expressed as (length × width^2^)/2. The tumor volume would be 100 nm^3^ at 20 days after inoculation.

Then, the animals were divided randomly into three groups again to receive different treatments, with 10 animals in each group, and there must be at least 2 model animals with A549, NCI-H460, and NCI-H446, respectively, in each treated group. The control group was treated with normal saline by gavage once a day for 10 days; the YQCTF group was treated with 200 mg/kg YQCTF by gavage, which was equal to 2 times of adult dose, once a day for 10 days; the Sorafenib group was treated with Sorafenib by gavage, before administration, and Sorafenib storage solution was prepared in a 1 : 1 ratio of polyoxy ethylene to castor oil and 95% ethanol, and the solution was diluted to 3 mg/mL and was given once a day for 10 days.

### 2.3. YQCTF Configuration

YQCTF was composed of 15 g rhizoma pinellinae praeparata, 30 g Gen-Seng, 15 g thunberg fritillary bulb, and 15 g Indian Iphigenia Bulb (purchased from the Pharmacy of the First Affiliated Hospital of Guangzhou University of Chinese Medicine). The above herbs are decocted in ultrapure water for two times. For the first time, 10 times of water was added for soaking for more than 1 h, boil it in high heat, and then continue to boil it with soft fire for 1 h. Sterile gauze was used to filter the obtained liquid and collect the preboiled liquid. For the second time, 8 times of water was added, boil it in high heat, then turn to low heat for 1 h, and the filtered preboiled liquid was collected. The filtrate obtained by combining the above two decoctions was concentrated to a crude drug content of 4.0 mg/mL of the liquid, and the liquid was separately packed and stored at -20°C and thaw before use.

### 2.4. Immunofluorescence Staining and HE Staining

*Immunofluorescence staining*: lung transplantation tumor tissue sections were placed in an oven for drying for 4 h and then removed, followed by dewaxed treatment in xylene for 2 times, lasting for 5 min each time. Then, they were immersed in anhydrous ethanol, 95% ethanol, 90% ethanol, 80% ethanol, and 70% ethanol for 5 min in each gradient of ethanol and were washed in distilled water, after which the PBS buffer was used for rinsing. After drying and slicing, primary antibody was added and they were kept at 4°C overnight. On the second day, they were washed with PBS for 3 times, 5 min each, and finally dried, after which secondary antibodies were added. The types of secondary antibodies were corresponding to the primary antibodies. The sections were incubated at room temperature in the dark for 1 h. Finally, they were rinsed with PBS for 3 times for 5 min each and then dried. DAPI was used for restaining, and the sections were incubated at room temperature for 10 min, rinsed with PBS for 3 times, and then dried and sealed with antifluorescence quenching assay.

*HE staining*: 4 *μ*m thickness of lung transplantation tumor tissue sections were prepared and were extracted and copied for HE staining. The specific operation was as follows: the paraffin sections were dewaxed with xylene solution, dehydrated with gradient alcohol for 5 seconds, and then washed with water. After 5-10 min of hematoxylin staining, the excess dye was washed away and the sections were acidified with hydrochloric acid and ethanol. After 3-5 min of eosin staining, the excess dye was washed away. The sections were dehydrated transparently with gradient ethanol for 5 s and dried overnight. Finally, the images were observed and photographed under the optical microscope, and the computer was used for subsequent processing.

### 2.5. Transmission Electron Microscopy Detection

Transplanted tumor tissue specimens were taken and cut into small cubes of 1 × 1 × 1 m^3^, which were quickly fixed in 2.5% glutaraldehyde solution, after which rinsed with 0.1 m phosphate for 3 times, each time lasting for 15 min. They were fixed in 50% ethanol, 70% ethanol, and 90% ethanol for 15 min, respectively. After drying overnight in an oven at 37°C, ultrathin slicer was used for slicing them and 3% uranium acetate was used for dyeing. After rinsing with double steam water, they were stained with lead citrate for 15 min and finally observed and photographed under transmission electron microscope.

### 2.6. Real-Time PCR Detection

The transplanted tumor tissue was regarded as samples, fluorescence quantitative kit (Genetimes Technology, China) was adopted in quantitative PCR (Thermo Fisher Scientific, USA) to conduct quantitative test on VEGFR gene, results showed that the calculation of the Tm value was greater than 60°C, and the dissolution curve was unimodal, so it was deemed that gene amplification was with specific gene. 2-*ΔΔ*Ct was used to represent the relative quantitative results. With GAPDH as the internal reference gene, VEGFR primer sequences were detected as follows: upstream primer F: 5′-TCGAGCCCTCATGTCTGAAC-3′ and downstream primer R: 5′-TGATGCTGTCCAAGCGTCTT-3′; primer sequence of internal reference GAPDH: upstream primer F: 5′-CTTAGCACCCCTGGCCAAG-3′ and downstream primer R: 5′-GATGTTCTGGAGAGCCCCG-3′.

### 2.7. Western Blot for Protein Expression Level Detection

According to the experimental operation of the kit, reagent A and reagent B were mixed in the 50 : 1 ratio and were shaken evenly and configured into BCA working liquid. After adding 2 *μ*L of the tested sample into each sample hole of the 96-well plates, PBS was added to make up to 20 *μ*L, and then, 200 *μ*L working fluid was added to each hole to be tested. After oscillation and blending, it was placed in an incubator at 37°C for 30 min and cooled at room temperature. Finally, the absorbance was detected at 562 nm, and OD value was determined by enzyme-linked immunosorbent assay (ELISA). The concentration of the protein in the sample was calculated according to the calculated standard curve and the dilution ratio of the sample in the test.

*Electrophoresis detection*: the extracted proteins were run by electrophoresis and transferred to the membrane in the SDS-PAGE gel. After sealed with 5% of the blocking solution and incubated at room temperature for 1 h, the sealed membrane was placed in the primary antibody, and the plate was shaken at room temperature for 10 min and left overnight at 4°C. The membrane was incubated with a secondary antibody at room temperature for 1 h. After washing the membrane for color development, the Image J software was used to analyze the gray scale of the protein bands.

### 2.8. Statistical Analysis

The SPSS 18.0 software was adopted for statistical analysis. The count data were expressed as mean plus or minus standard deviation (x¯±s), *t*-test was adopted for comparison between two groups, one-way ANOVA was adopted for comparison between multiple groups, and Dunnett's test was adopted for comparison between groups. *P* < 0.05 was considered statistically significant.

## 3. Results

### 3.1. Construction Results of Lung Cancer Subcutaneous Transplanted Tumor Model

Human lung adenocarcinoma model, human lung large-cell carcinoma model, and human lung small-cell carcinoma model were successfully constructed with A549, NCI-H460, and NCI-H446 cell lines, respectively. The site of transplanted tumor in rats of all groups was subcutaneous on the right back, and the appearance of rats of all groups was intact and neat. The results of HE staining of transplanted tumor tissues in each group are shown in Figure 1. A549 model tumor showed nests of cancer cells with enlarged nuclei, the cell morphology was abnormal, and the overall features were consistent with the pathological features of lung adenocarcinoma. NCI-H460 model tumor was observed under the microscope that the overall volume of cancer cells increased significantly and the cancer cells were round, the nucleus was enlarged and cytoplasm decreased, and the overall characteristics were consistent with the pathological characteristics of large-cell lung cancer. NCI-H446 model tumor had rounded and oval cancer cells under macroscope, cells were with rare cytoplasm and unclear cell boundaries, fine granular chromatin could be observed in the nucleus, the nucleus was absent or not obvious, and the overall characteristics were consistent with the pathological characteristics of small-cell lung cancer.

### 3.2. Growth of Lung Cancer Subcutaneous Transplanted Tumor Inhibited by YQCTF

The A549, NCI-H460, and NCI-H446 model rats were administered with YQCTF, positive drug Sorafenib, and normal saline once a day for 10 days, respectively. The results in Figure 2 showed that the YQCTF could inhibit the proliferation of all types of lung cancer transplanted tumors.

For the A549 model rats, the average tumor volume of the YQCTF-treated group was smaller than that of the control group from the 8th day, and the difference was statistically significant (*P* < 0.05), and the positive drug Sorafenib-treated group had the smallest average tumor volume and the best inhibitory effect. For the NCI-H460 model rats, the tumor inhibition effect of the YQCTF-treated group was more obvious, and it was observed that the average tumor volume of the YQCTF-treated group was smaller than that of the control group on the fourth day, and the difference was statistically significant (*P* < 0.05), and the inhibitory effect of the YQCTF-treated group was similar to the positive drug Sorafenib-treated group. For the NCI-H446 model rats, the YQCTF treatment also had a good inhibitory effect on the tumor, and it was significantly observed that the average tumor volume of the YQCTF-treated group was smaller than that of the control group on the fourth day, and the difference was statistically significant (*P* < 0.05), and the inhibitory effect of the YQCTF-treated group was even better than that of the positive drug Sorafenib-treated group. Calculation equation of tumor growth inhibition (TGI) was as follows. TGI = (1 − average tumor volume in the treated group/average tumor volume in the control group) × 100%. At the 10th day of intervention, the TGI of the A549 model rats treated with YQCTF and the Sorafenib were 42.3% and 65.0%, respectively; the TGI of the NCI-H460 model rats treated with YQCTF and the Sorafenib were 84.5% and 87.3%, respectively; the TGI of the NCI-H446 model rats treated with YQCTF and the Sorafenib were 56.9% and 49.2%, respectively, as shown in Figure 3. The volume changes of different transplanted tumors in different intervention groups are shown in Tables 1–3.

### 3.3. Effect of YQCTF on Angiogenesis of Lung Cancer Transplanted Tumor

Immunofluorescence staining of CD31 was performed on the tissue sections of different transplanted tumors, and the vascular endothelial structure was observed under the microscope. As shown in Figures 4 and 5, among the three kinds of lung cancer transplanted tumor groups, the vascular density in each group treated with YQCTF was significantly reduced compared with that in the control group (*P* < 0.05). The structures of lumen were also significantly lower than those of control group, which indicated that the YQCTF could not only inhibit the number of blood vessels, but also affected the morphological progression of blood vessels to a certain extent.

### 3.4. Effect of YQCTF on the Structure of Endothelial Cells of Angiogenesis in Lung Cancer Transplanted Tumor

The structure of angiogenesis endothelial tissues of lung cancer transplanted tumor tissues was observed under transmission electron microscope. The cell membrane of vascular endothelial tissues of the control group was intact and smooth, the cell structure was clear and complete, the nuclear morphology was normal, and the overall cell size did not increase or decrease, while the cell membrane of vascular endothelial tissues in the YQCTF-treated group showed obvious shrinkage, the overall morphology of the cells was not complete, the nucleus shrank, the nucleoli gathered under the nucleus, and the cytoplasm showed vacuolation, as shown in Figure 6.

### 3.5. Effect of YQCTF on the Expression of Angiogenesis-Related Molecules in Lung Cancer Transplanted Tumor

Vascular endothelial cells are the target of many proangiogenic factors, on which a variety of proangiogenic factor receptors are distributed. Endothelial cells themselves can also express cytokines that regulate angiogenesis, and these cytokines act on other adjacent endothelial cells in paracrine form. Western blot and quantitative PCR were adopted to observe the effect of YQCTF on the expression of proangiogenic factor or its receptor in vascular endothelial cells. After tumor exfoliating in each group, the total protein of nude rats was extracted and the protein expressions of VEGF, HIF-1, DLL4, and Notch-1 were detected. The protein changes of VEGF, HIF-1*α*, DLL4, and Notch-1 in each transplanted tumor group treated with YQCTF are shown in Tables 4–6 and Figure 7. In each transplanted tumor group, the protein levels of VEGF, HIF-1, DLL4, and Notch-1 in the YQCTF-treated group were significantly lower than those in the control group (*P* < 0.05), and the inhibitory effect of YQCTF treated group was similar to that of the positive drug Sorafenib-treated group. Quantitative PCR showed that the mRNA expression of VEGF in the transplanted tumor was inhibited by YQCTF, and the inhibitory effect was similar to or even greater than Sorafenib, as shown in Figure 8.

## 4. Discussion

The formation of angiogenesis is necessary for both tumor growth and metastasis, which plays an important role in the progression of many malignant tumors. How to control tumor angiogenesis is a top priority in many cancers, including lung cancer [12–14]. Traditional Chinese medicine believes that lung cancer mostly due to deficiency of vital “qi” and poison enters lung, making lung blocked, the metabolize is not free, phlegm is produced inside, the lung goes down for a long-time spittoon twine, and precipitate is formed or the spleen is weak, the metabolism is not free, and the moisture gathers and forms the phlegm dense lung. Therefore, the pathogenesis of lung cancer is closely related to phlegm and deficiency [15–18]. According to the theory of traditional Chinese medicine, the YQCTF had certain inhibitory effect on lung cancer, and it was found in this experiment that the growth of NSCLC and SCLC transplanted tumor could be effectively inhibited by it, and the effect was particularly excellent for large-cell carcinoma cancer and small-cell carcinoma cancer, which was similar to the results obtained in vivo by Janghorban et al. [19]. In this experiment, it was also found that the YQCTF could not only reduce the number of tumor angiogenesis, but also improve the formation of tumor angiogenesis lumen and did well in both large-cell and small-cell carcinomas. According to speculation of Jakovljevic et al., it may be related to the DLL4-Notch signaling pathway [20]. DLL4-Notch signaling pathway was currently considered to have the highest correlation with tumorigenesis, especially tumor angiogenesis, which was highly expressed in many tumors, including lung cancer [21–23]. The results of this experiment showed that DLL4 and Notch were highly expressed in all nude rats with lung cancer transplanted tumor and decreased to a certain extent after treatment with YQCTF. Combined with the size of subcutaneous graft tumor, further results could be obtained that DLL4 and Notch were associated with the characterization and size of tumor to some extent. Borghetti et al. also suggested that DLL4 and Notch had similar effects on the progression of lung cancer [24]. In the experiment, it was found that under the action of the YQCTF, the angiogenesis appeared shrinkage and the degree of shrinkage was more obvious, which further demonstrated the mechanism of inhibiting tumor growth by acting on DLL4 and Notch on angiogenesis. In clinical, YQCTF has played a certain role in the treatment of lung diseases, for it was believed that the clinical trial of YQCTF for the treatment of lung cancer is safe and feasible.

## 5. Conclusion

In this study, different types of lung cancer transplanted tumor models were constructed, the effects of YQCTF on lung cancer growth and angiogenesis were observed in vivo, and the effects on the expression of VEGF, DLL4-Notch signaling pathway, and related factors in lung cancer tissues were analyzed. The results showed that YQCTF mainly inhibited the proliferation of lung cancer transplanted tumors by inhibiting the angiogenesis in lung cancer tissues, reduced the number of angiogenesis, and destroyed the lumen structure of angiogenesis. VEGF signaling pathway and DLL4-Notch signaling pathway were downregulated to destruct the lung cancer angiogenesis. The experiment confirmed that the YQCTF had certain inhibitory effect on the growth of lung cancer and the angiogenesis of lung cancer, which provided a theoretical basis for the clinical application of the YQCTF in the treatment of lung cancer. However, as lung cancer and lung cancer angiogenesis were regulated by various vascular factors, further experiments and studies were required on more mechanisms of the effect of the YQCTF on lung cancer.

## Figures and Tables

**Figure 1:** HE staining results of transplanted tumor tissue sections of each group.

**Figure 2:** Inhibition effect of YQCTF on growth of three lung cancer transplanted tumor groups.

**Figure 3:** Changes of tumor volume in different treated rats ((a) A549 model rats; (b) NCI-H460 model rats; (c) NCI-H466 model rats).

**Figure 4:** Fluorescence staining results of lung cancer transplanted tumor tissue sections.

**Figure 5:** Quantitative results of angiogenesis.

**Figure 6:** Effects of YQCTF on ultrastructure of angiogenesis endothelial cells of lung cancer transplanted tumor in each group.

**Figure 7:** Expression of VEGF, HIF-1, DLL4, and Notch-1 protein in each transplanted tumor group treated with YQCTF ((a) A549 model rats; (b) NCI-H460 model rats; (c) NCI-H466 model rats).

**Figure 8:** Comparison of the effects of YQCTF on the mRNA expression level of VEGF in each lung cancer transplanted tumor group.

**Table 1:** Changes in volume of implanted lung adenocarcinoma after different interventions.

Time	Control volume (mm^3^)	YQCTF volume (mm^3^)	Sorafenib volume (mm^3^)
0 d	100.2 ± 8.0	103.3 ± 11.4	104.0 ± 9.4
2 d	125.4 ± 11.1	121.6 ± 13.6	123.4 ± 13.6
4 d	332.8 ± 19.7	178.9 ± 14.2	142.6 ± 15.1
6 d	397.4 ± 19.2	231.1 ± 24.3	133.2 ± 14.8
8 d	494.9 ± 23.8	298.5 ± 33.6	156.7 ± 11.9
10 d	773.9 ± 41.3	399.3 ± 40.4	198.3 ± 20.2

**Table 2:** Changes in tumor volume of implanted large cell tumor after different interventions.

Time	Control volume (mm^3^)	YQCTF volume (mm^3^)	Sorafenib volume (mm^3^)
0 d	87.1 ± 7.5	89.3 ± 6.4	86.8 ± 5.3
2 d	497 ± 24.1	100.5 ± 7.6	103.1 ± 10.3
4 d	521 ± 26.7	103.9 ± 7.4	105.7 ± 11.7
6 d	998 ± 56.4	187.3 ± 12.5	188.2 ± 15.3
8 d	1442 ± 60.2	176.8 ± 11.6	179.5 ± 16.8
10 d	2014 ± 76.5	180.6 ± 15.8	181.7 ± 15.3

**Table 3:** Changes in the volume of implanted small cell tumor after different interventions.

Time	Control volume (mm^3^)	YQCTF volume (mm^3^)	Sorafenib volume (mm^3^)
0 d	100.2 ± 8.3	102.1 ± 6.6	103.6 ± 7.9
2 d	111.4 ± 7.2	104.9 ± 10.1	106.3 ± 8.4
4 d	197.1 ± 14.9	111.0 ± 11.6	112.2 ± 12.3
6 d	225.8 ± 16.2	125.7 ± 9.8	135.7 ± 9.6
8 d	354.9 ± 21.0	131.5 ± 8.3	142.2 ± 13.8
10 d	467.3 ± 24.6	142.3 ± 13.4	155.8 ± 15.9

**Table 4:** Expression levels of related proteins in A549 model rats.

Group	VEGF expression	HIF-1 expression	DLL4 expression	Notch-1 expression
Control	100.31 ± 9.93	100.03 ± 5.49	100 ± 15.23	100.01 ± 4.49
YQCTF	57.99 ± 4.19	69.66 ± 5.14	13.79 ± 4.25	55.91 ± 7.316
Sorafenib	54.23 ± 4.32	65.23 ± 5.47	11.87 ± 4.56	52.32 ± 7.14

**Table 5:** Expression levels of related proteins in NCI-H460 model rats.

Group	VEGF expression	HIF-1 expression	DLL4 expression	Notch-1 expression
Control	98.21 ± 5.21	97.41 ± 6.32	96.09 ± 2.44	99.42 ± 6.52
YQCTF	56.87 ± 3.65	68.32 ± 5.64	14.39 ± 2.65	54.97 ± 2.65
Sorafenib	54.51 ± 6.54	66.32 ± 2.56	10.32 ± 5.12	51.78 ± 6.45

**Table 6:** Expression levels of related proteins in NCI-H446 model rats.

Group	VEGF expression	HIF-1 expression	DLL4 expression	Notch-1 expression
Control	98.29 ± 5.12	96.22 ± 6.98	95.87 ± 5.65	96.05 ± 5.64
YQCTF	66.32 ± 2.45	71.23 ± 3.65	23.36 ± 3.45	62.32 ± 5.87
Sorafenib	62.75 ± 6.32	68.32 ± 7.925	20.12 ± 5.64	59.32 ± 2.32

## Data Availability

Some or all data, models, or code generated or used during the study are available from the corresponding author by request.
